The article "Evaluation of SDS‐coated iron nanostructure on the gene expression of bio surfactant‐producing genes by Pseudomonas aeruginosa" was retracted in 2025. Reasons: manipulated images; plagiarized images; overlap with other authors' work; compromised peer review.

# Evaluation of SDS‐coated iron nanostructure on the gene expression of bio surfactant‐producing genes by *Pseudomonas aeruginosa*

**DOI:** 10.1002/elsc.202200002

**Published:** 2022-08-24

**Authors:** Yaser Ahsani Arani, Zahra Noormohammadi, Behnam Rasekh, Fatemeh Yazdian, Hojjat kazemi

**Affiliations:** ^1^ Department of Biology Science and Research Branch Islamic Azad University Tehran Iran; ^2^ Environment & Biotechnology Research Division Research Institute of Petroleum Industry (RIPI) Tehran Iran; ^3^ Department of Life Science Engineering Faculty of New Science and Technologies University of Tehran Tehran Iran; ^4^ Analytical Chemistry Research Group Research Institute of Petroleum Industry (RIPI) Tehran Iran

**Keywords:** bio surfactant, Fe/SDS nanoparticle, gene expression, *Pseudomonas aeruginosa*

## Abstract

Bio surfactants are natural surfactants that induce emulsification, displacement, increased solubility, and mobility of hydrophobic organic compounds. In this study, the gene expression of biosurfactant production genes by *Pseudomonas aeruginosa* in the presence of sodium dodecyl sulfate coated iron nanostructure (Fe/SDS) were evaluated. Emulsification Index and Surface Tension reduction test to check stability and emulsification the rhamnolipid were done. Purification was evaluated using thin layer chromatography (TLC) and expression of *rhlA*, *mvfR, lasR, rhlR* genes was determined using q‐PCR technique. Binding of nanoparticles to bio surfactants was confirmed by TEM. The best emulsification index, was by the sample that exposed to 1 mg/L Fe/SDS nanoparticles for 2 days. Rhamnolipid produced in the presence of nanoparticles had an acceptable ability to reduce surface tension. The Rf (retention factor) value obtained was 0.63 by chromatography. q‐PCR results showed that the expression *of rhlA, mvfR, lasR, rhlR* genes was significantly increased in Fe/SDS treated cells, which indicates the significant positive effect (*P* < 0.05) of nanoparticles on biosurfactant production of treated cells. While, SDS and Fe alone were not affected significantly (*P* > 0.05) on the expression of these genes. Our findings indicated the importance of nanoparticles in increasing the expression of genes involved in the bio surfactant production pathway of *Pseudomonas aeruginosa*.

**Abbreviations**
Fe/SDS: sodium dodecyl sulfate coated iron nanostructure
QS: quorum sensing
qPCR: quantitative polymerase chain reaction
SDS: sodium dodecyl sulfate
SEM: scanning electron microscope
TEM: transmission electron microscopy
TLC: thin layer chromatography

## 1 INTRODUCTION

Some microorganisms in nature are able to secrete extracellular substances, including various enzymes and biosurfactants. Biosurfactants are surface‐active molecules [1, 2]. Development of biosurfactants and their commercialization have increased significant in recent years [3]. Biosurfactants are unique amphiphilic compounds that have both hydrophobic and hydrophilic components, therefore increase the bioavailability of water in the compounds and alter the bacterial cell wall. Surface activity has turned these materials into excellent emulsifiers [4, 5]. Bio surfactants are one of the most important products of industrial microbiology and are produced by bacteria, fungi and yeasts in stationary phase [6]. Some characteristics of bio surfactants that make them superior to chemical surfactants include: reduction of surface and interfacial tension, low toxicity, high biodegradability, emulsification, selective performance, specific activity, possibility of production from cheap raw materials, antimicrobial properties, easier production and more variety [7, 8].

The reduction in the surface tension of the culture medium indicates the production of surfactants by bacterial cultures and has been shown to contribute to substrate metabolism [9]. The main application of bio surfactants is in petroleum industry which are used in oil purification and decontamination of organic compounds, increasing the bioavailability of these compounds, removing contaminants with increasing solubility and emulsification during purification, removal of residual oil from storage tanks, enhancing oil recovery and soil and water bioremediation [10].

Rhamnolipids are one of the most important glycolipid bio surfactants, which are produced by two bacterial species of *Pseudomonas Aeruginosa* and *Burkholderia* [11]. Ramnolipid has a high emulsion capacity and is often used in the pharmaceutical and environmental industries such as increasing oil recovery and bioremediation [12]. *Pseudomonas* species are the largest producers of rhamnolipids. *Pseudomonas* is one of the most important soil bacteria that can break down polycyclic aromatic hydrocarbons to produce rhamnolipids, quinolones, hydrogen cyanides and lectins, indicating the microorganism's inherent resistance to a variety of chemicals [13]. Also *Pseudomonas aeruginosa* is one of the most important Infectious agents [14]. *Pseudomonas aeruginosa* produces two different types of rhamnolipids that differ in the number of rhamnose sugars. Mono‐rhamnolipids and di‐rhamnolipids are the main rhamnolipids. These molecules have high surface activity and are used in various medical fields as antifungal, antibacterial and antiviral materials. Other application of rhamnolipids in the oil industry is in microbial enhanced oil recycling and removal of oil contaminants from the environment, as well as cleaning tankers and facilitating crude oil transportation [13]. The limitation of using rhamnolipid for cleaning of oil tanks is the separation of bio surfactants.

One of the methods of recycling and separation of bio surfactants is the use of magnetic iron nanoparticles [15]. Nowadays, study of the effects of metal nanoparticles on bacterial growth and production of bio surfactants has gained a great attention. One of the recent studies showed the antibacterial properties for some types nanoparticles by physical destruction of the cell wall or oxidative stress, while there are several types of nanoparticles that have significant positive effects on bacterial growth, possibly due to their higher specific surface area and ability to release electrons [16]. Some of the nanoparticles in certain concentrations not only don't have antimicrobial effects, but also they increase the level of bacterial contact with the compounds in the culture medium and further exchange of nutrients and thus increase the production of bio surfactants. The results of these studies vary depending on the type of bacteria, type of nanoparticles, concentration of nanoparticles, and duration of interaction of nanoparticles with bacteria [16].

**PRACTICAL APPLICATION**

This research is the use of Fe/SDS nanoparticles in production of bio surfactant and increasing gene expression involved in the production of bio surfactant from *Pseudomonas aeruginosa*.

The effect of Fe nanoparticles and their derivatives, such as iron oxide or coated iron nanoparticles, on various bacterial processes, such as bacterial growth rate, has been studied. The coating of Fe nanoparticles is often performed to reduce oxidizing power of these nanoparticles. [17, 18]. Rezazadeh et al. investigated the production of bio surfactant by *Pseudomonas aeruginosa* using iron/starch nanoparticles. In this study, starch‐coated iron nanoparticles did not show any bacterial toxicity at 1mg/ml and increased the growth rate and production of bio surfactants to 20.62% [19]. Modabber et al., was investigated the effect of starch coated Fe^0^ and Fe^3+^ nanoparticles on the production of surfactin from *Bacillus subtilis* [20]. The expression of most *Pseudomonas aeruginosa* genes is controlled by the Quorum sensing (QS) gene system. According to the genetic pathway of bio surfactant synthesis in *Pseudomonas aeruginosa* and its relationship with QS signaling pathway, genes related to bio surfactant production include *rhl A, rhl B, lasR/I, rhlR/I, pqsR/pqsA* [21]. QS is a cell‐to‐cell communication system using small signaling molecules in single‐celled organisms [22]. In *Pseudomonas* bacteria, the QS system consists of two gene systems, *LasI‐LasR* and *RhlI‐RhlR*. The *LasI* and *RhlI* genes synthetize two enzymes (HSL‐acyl) (lactone hemoserine‐a), while the *LasR* and *RhlR* produce transcriptional regulatory proteins that bind to their own signal to activate genes [23]. The *lasI* gene regulates the production of elastase, exotoxin A and alkaline protease, while the *rhlI* gene is responsible for regulating the production of rhamnolipid, alkaline protease, elastase and cyanide [24].

Despite the ecological importance of *Pseudomonas aeruginosa* bio surfactant, rare researches have been reported on the effect of nanoparticles on the genes regulating the production of this bio surfactant and their related control systems. The sodium dodecyl sulfate coated iron (Fe/SDS) as iron nanoparticle were used in present study. SDS was chosen as a coating for iron nanoparticles due to the wide application of this detergent in industries related to the removal of oil pollution from the environment, especially soil [25]. The aim of this study was 1‐ to evaluate gene expression profile involved in the production and, 2‐ to survey the regulation of *Pseudomonas aeruginosa* bio surfactant production in the presence of Fe/SDS nanoparticles.

## 2 MATERIALS AND METHODS

### 2.1 Materials

Fe/SDS nanoparticles were purchased from Zist‐Tajhiz Pars Company, Tehran, Iran and the effect of nanoparticle on bacteria was investigated at a concentration of 1 mg/L. PBS buffer was used (pH 7.4, KH_2_PO_4_ 0.27 g/L, Na_2_HPO_4_⋅2H_2_O 1.78 g/L, KCl 0.2 g/L, Nacl 8.01 g/L) [26].

### 2.2 Microorganism

*Pseudomonas aeruginosa* PBCC5 was used. It was prepared from petroleum biotechnology culture collection (WDCM 964) of the Research Institute Petroleum Industry (RIPI). It is Gram‐negative and rod‐shaped and Gram‐negative Bacterium by diagnostic methods and microscopic observation by the naked eye, after 48 h of incubation in nutrient agar medium.

### 2.3 Preparation of bacterial growth curve in molasses culture medium

The molasses used in this research were prepared from Marvdasht Sugar Factory in Shiraz. Two types of culture medium, liquid nutrient culture medium for overnight culture and molasses culture medium 15% (w/v) were prepared as the main culture medium for growth and production of *rhamnolipid*. The ambient pH was raised to 7 by 1M HCl and sterilized by autoclave [27]. To prepare the bacterial growth curve, after preparing the overnight culture, microbial inoculation was performed on the molasses medium and every 2 h in sterile conditions, 2 ml of the culture medium was sampled and bacterial growth was measured based on cell density using spectrophotometer at 600 nm [28], In several studies, nanoparticles increase the growth of microorganisms by decreasing the lag phase and increasing the logarithmic and Stationary phase, for this purpose, they are added to the bacterial culture medium at the beginning. In this study, nanoparticles were inoculated into the bacterial culture medium at the end of the Lag phase.

### 2.4 Emulsification activity (E_24_)

This test is to check the stability and emulsification of the sop from the bacteria after 24 h. Within 1 tube, 2 ml gas oil and 2 ml of supernatant with a volume ratio of 1:1, was poured. The sample was exposed to severe vortexed for 2 min. The samples were then kept for 24 h stabile and the emulsification activity (E_24_) were calculated after 24 h using the following formula: This test was done in three repetitions [29, 30].

(1) $$E_{24}=\frac{Height\;of\;emulsion\;layer}{Height\;of\;total\;liquid}\;\times 100$$

### 2.5 Surface tension measurement

Twenty‐five milliliter of 96 h culture of each sample were centrifuged at 10,000 rpm for 20 min, in order to remove the cells. Then surface tension was measured by tension meter (FTM‐TN‐556, Toos Nano). An effective bio surfactant can decrease the surface tension of water from 72 to 35 mN/m. This test was done in three repetitions [31].

### 2.6 Fe/SDS nanoparticle

Four Erlenmeyer flasks (250 ml) containing 50 mL of 15% sterile molasses culture medium with Fe/SDS nanoparticles at a concentration of 1 mg/L, Fe at a concentration of 1 mg/l, SDS at a concentration of 1 mg/L and no additive as control sample were used.

SEM (KYKY_EM3200 model) was used to ensure the placement of nanoparticles on the bacterial surface and to examine the morphology of the surface. For this purpose, 25 μl of the sample was poured onto a slide and the solution was dried in the presence of air. The samples were coated with gold for a few seconds to make them conductive. Then, the surface morphology was examined by SEM.

### 2.7 Gene expression assay

In this research Genes expression *rhlA mvfR*, *lasR, rhlR* genes by RT PCR reaction were investigation. To study gene expressions, RNA was extracted from cells by RNX‐PLUS. Treated cells were cultured for 72 h and were centrifuged, then 500 μL RNX‐PLUS solution was added to the cell sample and vortexed for 5 s. Then, 200 μL chloroform was added. The resulting mixture was centrifuged at 12,000 g for 15 min at 4°C, and was placed in the freezer for 30 min, the supernatant was discarded and 1 mL of 75% ethanol was added and centrifuged for 8 min at 4°C and the mixture was allowed to dry. Then, water 50°C was added. RNA concentration was measured by optical density method using Nano drop device. RNA was evaluated at 280 and 260 nm.

A bio Fact kit (bio Fact, Korea) was used for cDNA synthesis according manufacturer protocol. In order to make cDNAs, a volume equivalent to 1000 ng was used. The final volume was 20 Landa. In a free RNase micro type, 10 μL 2X RT Pre‐Mix, 10 ng–5 μg Total RNA, 1 ng–0.5 μg mRNA, Primer (Oligo (dT) 20:50, Random Hexamer 50 μM, Sequence‐Specific Primer 15–20 μM) and for the remaining volume up to 20 Landa, water was added to each sample. The micro tubes were placed in a thermo cycler for 5 min at 37°C, 30 min at 50°C and 5 min at 95°C, and cDNA was synthesized during the set time.

The qPCR reaction was performed for quantitative analysis of gene expression by cyber green method using Corbett device. The materials required to perform the PCR reaction Include: cDNA samples, DNA ase and RNAase free Water, Taq DNA Polymerase Master Mix RED (Amplicon), Forward Primer, Reverse Primer were used.

Primer design was done using Primer 3 program. The thermodynamic properties and three‐dimensional shape of the primers were checked with Gene runner software. The primers designed for the genes are according to Table 1.

**TABLE 1:** Sequence of primers used in *Pseudomonas aeruginosa*

Name	Forward or reverse	Sequence (5′ → 3′)	Length
*rhlA*	F	ACATTTCAACGTGGTGCTGT	20
	R	GTGATTGACCTCGAAGCGC	19
*mvfR*	F	AAACTTCGACGACATGCTGC	20
	R	TCGTAGAGTTCGCTGAGGAC	20
*lasR*	F	CTTCGAACATCCGGTCAGC	19
	R	AGTTCACATTGGCTTCCGAG	20
*rhlR*	F	CTGGGCTTCGATTACTACGC	20
	R	TCTGCATCTGGTATCGCTCC	20
16S rRNA	F	TCGGACCTCACGCTATCAGA	20
	R	CCGTGTCTCAGTTCCAGTGT	20

Reaction temperature cycle of PCR is as follows: primary denaturation at 94°C for 5 min, double strand opening at 94°C for 1 min, primer binding at binding temperature of 52°C for 1 min, polymerization at 72°C for 90 s and final elongation at 72°C for 10 min [32].

### 2.8 Partial purification of rhamnolipids

The rhamnolipids were recovered by solvent extraction. Cell‐free supernatant was obtained by centrifugation of olive oil broth at 6000 rpm and 4°C for 15 min. The supernatant was acidifying to pH 2 using 6 N HCl and was incubated overnight at 4°C. Then, the supernatant was mixed with chloroform and methanol (2:1), and the organic layer was separated and dried at 40°C within 5–6 h [31].

### 2.9 Thin layer chromatography (TLC)

Thin layer chromatography was used to determine the number of compounds and active ingredients. In order to perform TLC, 60 silica paper with dimensions of 15×5 Cm was arranged. 0.1 mg of dried bio surfactant was dissolved in 10 μl of 90% ethanol and 5 μl of samples were dotted at a distance of 1Cm from the edge of the paper. The mobile phase consisting of chloroform, methanol, and acetic acid with a ratio of 2/15/65 v/v/v was selected. For staining, the solution containing 0.15 orcinol and 8.2 ml of 60% sulfuric acid in 42 ml of distilled water was sprayed on paper and dried at 140°C for 10 min.

Rf (retention factor) is a measure of the velocity at which a substance moves in a chromatographic system. The value of Rf, due to its uniqueness in each compound, can be used to identify compounds. When comparing two different compounds under the same conditions, a compound with a larger Rf value has less polarity. To determine Rf, the distance traveled by the object from the starting line to the middle of the stain is measured and divided by the distance traveled by the solvent. This distance is measured with the same starting line [33].

### 2.10 Data analysis

One‐way ANOVA statistical test was performed to compare the significant difference the values obtained from the expression of the desired genes between the study groups at the statistical level of 5% and Duncan multivariate test at the level of 1%. Values ​​less than 0.05 were considered significant. Statistical Data analysis was performed by SPSS 22 software.

## 3 RESULTS

Figure 1 shows the growth curve obtained from *Pseudomonas aeruginosa PBCC5*. According to the growth curve, the bacterium leaves the Lag phase at the 10th hour of its growth and enters the logarithmic phase, and the bacterial stationary phase begins at the 28th hour, when rhamnolipid production takes place at this stage.

**FIGURE 1:** (A) Growth curve of *Pseudomonas aeruginosa* PBCC5 in molasses culture medium. (B) Growth curve of *Pseudomonas aeruginosa* PBCC5 in molasses culture medium after addition nanoparticles

### 3.1 Emulsification index test (E_24_)

Emulsification index test was used to check stability and emulsification the rhamnolipid after 24 h. Emulsification activity was measured daily (24, 48, 72, and 96 h). Emulsification was not observed in any of the samples on the first day (24 h). On the second, third and fourth day (48, 72, 96, h), all samples had foam from the rhamnolipid emulsion, which indicated the onset of rhamnolipid production from 48 h after bacterial growth. From 48 to 96 h, the bio surfactant production was increased.

Emulsification indexes reduced with increasing the concentration of Fe/SDS nanoparticles from 500 to 1000 mg/l compared with control sample on the second day (48 h) while for sample exposed to 1 mg/l Fe/SDS, the emulsification index was higher than for control sample.

It is likely that this concentration of Fe/SDS (1 mg/l) causes bacteria to reach stationary phase sooner and produce biosurfactant. Any changes in emulsification indexes were observed on fourth day (96 h). According to the results of E_24_, it can be said that the low concentration of Fe/SDS (1 mg/l) nanoparticles caused the bacteria to reach stationary phase sooner and enhanced production of biosurfactant, while higher concentrations of nanoparticles (500, 1000 mg/l) decreased biosurfactant production in the first 48 h (Figure 2).

**FIGURE 2:** Effects of Fe/SDS nanoparticles on emulsification activity (E_24_)

In the present research, all samples had good emulsification activity in all days, but the best emulsification index, was by the sample that exposed to 1 mg/l Fe/SDS nanoparticles for 2 days, because of the faster *rhamnolipid* production in this sample.

### 3.2 Surface tension reduction test

Surface tension reduction of samples was measured after 96 h of incubation and were compared to water surface tension (72 mN/m). The results showed samples had the surface tension less than 40 mN/m and were reduced the surface tension of distilled water from 72 to 33–35.5 mN/m. In the similar study, by Alamdar et al. Effects of Fe/SDS and Au nanoparticles on *Pseudomonas aeruginosa* bacterial growth and biosurfactant production were examined. All samples, the surface tension of distilled water decreased from 72 to 32–35 mN/m [35].

The results showed that all samples decreased the surface tension from 72 of distilled water to 32–35 mN/m. According to these results, it was demonstrated that Fe/SDS nanoparticles at different concentrations did not have a negative effect on surface tension (Figure 3).

**FIGURE 3:** Effect of Fe/SDS nanoparticle concentration on the surface tension of biosurfactants after 96 h of incubation

### 3.3 Morphology of Fe/SDS nanoparticles with bacteria

SEM image of the Fe/SDS nanoparticles is provided in Figure 4. According to the image, the nanoparticles were spherical in shape and had an average size of 20 nm.

**FIGURE 4:** SEM image of Fe/SDS nanoparticles

Transmission electron microscopy (TEM) image (Figure 5) showed the placement of nanoparticles on the surface and membrane of bacteria. Nanoparticles in different concentrations increase the exchange of bacterial nutrients with the culture medium by increasing the bacterial surface and thus increase the growth and production of biosurfactant. Exposure of Fe/SDS nanoparticles to *Pseudomonas aeruginosa PBCC5* was performed at the beginning of the bacterial growth phase at a concentration of 1 mg/l and the results were compared with a control sample (without the presence of nanoparticles).

**FIGURE 5:** TEM image of bacteria in the presence of Fe/SDS nanoparticles

### 3.4 Expression of *mvfR, lasR, rhlR, rhlA* genes

Our findings showed that *rhlA* gene expression was significantly increased (*P* = 0.0001) in Fe/SDS treated cells (Figure 4), indicating the strong effect of this nanoparticle on the biosurfactant production of treated cells. However, SDS and Fe particles treatments alone were not effective in expressing the *rhlA* gene and were almost identical to the control sample.

The expression of *lasR, rhlR* and *mvfR* genes was also significantly increased (*P* = 0.0004, *P* = 0.005, *P* = 0.0001, respectively) in Fe/SDS‐treated cells, indicating the positive effect of nanoparticle on the treated cells. No significant effects were reported in *lasR* gene expression in SDS as well as Fe treated cells separately (Figure 6). Table 1 shows the analysis of variance of *mvfR, lasR, rhlR, rhlA* genes.

**FIGURE 6:** Expression of *lasR(A)*, *rhlA(B)*, *mvfR(C)*, *rhlR(D)* genes by RT‐PCR method in Fe/SDS treated cells

Based on analysis, all four genes, the means of gene expression levels in cells treated with Fe/SDS nanoparticles showed significant differences (Table 1), while SDS and Fe nanoparticles separately treatments showed no significant difference in the expression of *mvfR, lasR, rhlR* and *rhlA* genes (*P* = 0.0001, *P* = 0.0004, *P* = 0.005, *P* = 0.0001). the analysis indicated the importance of nanoparticles in increasing the expression of genes involved in the production of bi osurfactant from *Pseudomonas aeruginosa*.

### 3.5 Thin layer chromatography (TLC)

Thin layer chromatography was used to confirm the presence of biosurfactant from *Pseudomonas aeruginosa*. Rf (retention factor) was determined by the ratio of the distance traveled by the produced bio surfactant to the distance traveled by solvent. The Rf value obtained from TLC was 0.63 (Figure 7).

**FIGURE 7:** Thin layer chromatography (TLC)

## 4 DISCUSSION AND CONCLUSION

The most of expression genes in *Pseudomonas aeruginosa* are controlled by a gene system called the QS system. Today, several studies have been conducted to study the effects of metal nanoparticles on the growth of bacteria and the production of bio surfactants in various industrial fields. The results of these studies varied depending on the type of bacteria, the type of nanoparticles and the concentration of nanoparticles. Alamdar et al., reported the effect of Fe/SDS and Au nanoparticles on the growth and production of biosurfactant from *Pseudomonas aeruginosa PBCC5* [35]. Sahebnazar et al. used iron‐silica nanoparticles in molasses culture medium to increase the growth of *Pseudomonas aeruginosa* and increase the production of rhamnolipid [27]. In another study, the effect of nanoparticles on the expression of bacterial genes was investigated. The results showed an increase in the expression of some genes at specific concentrations of nanoparticles. Therefore, in addition to increasing bacterial surface in the presence of nanoparticles, nanoparticles may increase the expression of some genes involved in the bacterial growth and production of bacterial bio surfactants [15]. In this study, the expression of genes involved in the production of biosurfactant by *Pseudomonas aeruginosa* in the presence of Fe/SDS nanoparticles was investigated. At the first, in order to evaluate the efficiency of rhamnolipid produced, surface tension test and Emulsification activity (E_24_) were performed, which shows the proper performance of rhamnolipid in the presence of nanoparticles. In the study of Bendaha et al, emulsification index of bio surfactant produced by Pseudomonas aeruginosa PBCC5 for sample of 1 mg/l Fe/SDS, was reported at the second day of incubation [34], Which was consistent with the data in our research. Also, EI‐Sheshtawy reported that the most biosurfactant production by Bacillus licheniformis happen after 72 h, and their bio surfactants were secondary metabolites [31]. The results show that, rhamnolipid produced by *Pseudomonas aeruginosa* in the presence of nanoparticles, has an acceptable ability to reduce surface tension and can be used as a natural emulsifier in the oil industry. Expression of *rhlA, mvfR, lasR, rhlR* genes was evaluated using RT‐PCR and TLC chromatography. Data were analyzed by SPSS_22_ software and the means were compared based on ANOVA at 5% level and Duncan multivariate test at 1% level.

RT‐PCR results showed that the expression of *rhlA, mvfR, lasR, rhlR* genes was significantly increased in Fe/SDS treated cells, which indicates the positive effect of nanoparticles on treated cells. While SDS and Fe alone were not effective in the expression of these genes and were similar to the control sample.

According to the results, the highest and lowest gene expression in the presence of Fe/SDS nanoparticles belonged to *lasR* gene and *mvfR* gene, respectively. Statistically, the expression of *mvfR, lasR, rhlR* and *rhlA* genes were significantly increased in Fe/SDS‐treated cells. In a similar study, the frequency of quorum genes was reported to be 43.3%, 63%, 3.71%, and 3% for *laslI, rhlR, lasI* and *lasR* genes, respectively [27], In the study of *Senturk* et al., four isolates had *lasR, lasI, rhlR* and *rhlA* genes. One of the isolates lacked *lasR* gene and one isolate had none of the three *lasR*, *lasI* and *rhlR* genes [36]. Deficiency in the production of QS genes can be due to the production of extracellular enzymes that lead to the breakdown of genes encoding quorum sensing [36]. Another reason for the difference in the expression of QS genes may be due to point mutations in the genes encoding the QS system. Bjarnsholt et al. found that increased mutations in point mutations genes led to functional defects in *lasR* and *rhlR* genes [37]. The presence of several strains of *Pseudomonas aeruginosa* at the site of infection may lead to a defect in the expression of genes encoding the QS system [36].

The reason for this difference in the expression of QS genes and its association with drug resistance in *Pseudomonas aeruginosa* isolates requires further research. Due to the presence of different genes in *Pseudomonas aeruginosa* and due to the main role of QS genes, the frequency of these genes is not well defined and has been reported differently in various studies around the world.

In this research, according to the statistical results, *P*‐value <0.05 was obtained in all 4 genes for cells treated with Fe/SDS nanoparticles, which indicates the importance of nanoparticles in increasing gene expression involved in the production of bio surfactant from *Pseudomonas aeruginosa*.

## CONFLICT OF INTEREST

The authors certify they have no affiliations with or involvement in any organization or entity with any financial interest.

## Data Availability

All data generated or analyzed during this study are included in this article.
